This article has been retracted.

# Correlation and Diagnostic Value of Serum RBP4 and sRAGE and the Condition of Patients with Chronic Kidney Disease

**DOI:** 10.1155/2021/6166528

**Published:** 2021-10-27

**Authors:** Shihong Xiong, Ting Qi, Na Gong, Cheng Yang

**Affiliations:** ^1^Department of Nephrology, Tianyou Hospital Affiliated to Wuhan University of Science and Technology, Wuhan, Hubei 430064, China; ^2^Department of Nephrology, Puren Hospital Affiliated to Wuhan University of Science and Technology, Wuhan, Hubei 430081, China; ^3^Department of Gerontology, Hubei Hospital of Integrated Traditional Chinese and Western Medicine, Wuhan, Hubei 430015, China; ^4^Department of Nephrology, Central Theater General Hospital of PLA, Wuhan, Hubei 430070, China

## Abstract

Chronic kidney disease (CKD) is a progressive damage of renal structure and function caused by various reasons. Its course is long and irreversible. CKD can be divided into 5 stages according to the glomerular filtration rate (GFR). Early detection and early intervention of CKD can reduce the complications of patients and improve the survival rate. Retinol-binding protein 4 (RBP4) is a small molecule transporter. Receptor for advanced glycation end products (RAGE) is a multi-ligand transmembrane signal transduction receptor discovered in recent years. Soluble RAGE (sRAGE) is a new splicing heterogeneity of RAGE. Our results show that serum RBP4 is increased while sRAGE is decreased in CKD patients, both of which are closely related to the severity of CKD. The combined use of serum RBP4 and sRAGE has a high diagnostic value for CKD and can provide a reliable diagnostic basis for the clinic.

## 1. Introduction

Chronic kidney disease (CKD) is a chronic kidney injury caused by various causes of primary glomerulonephritis, secondary glomerulonephritis, diabetes, and hypertension. The main feature is the progressive deterioration or irreversible damage to the structure and function of the kidney [1]. In the early stages of CKD, patients may have no symptoms or only mild fatigue, low back pain, and nocturia. If left undiagnosed and untreated, as the disease progresses, it will eventually progress to stage 5 of CKD, known as end-stage renal disease (ESRD). ESRD patients have significantly reduced renal function and toxins accumulate in the body. It can cause symptoms such as loss of appetite, pruritus, and edema, as well as complications such as anemia and hypertension [2–4]. Therefore, it is important to actively treat CKD and delay its progression. Retinol-binding protein 4 (RBP4) is a transporter protein of retinol in the blood and is often present in the blood as a complex. It can induce insulin resistance by regulating fatty acid metabolism in the liver and muscle, leading to diabetes and its complications [5, 6]. Receptor for advanced glycation end products (RAGE) is one of the multi-ligand cell surface immunoglobulin superfamilies of receptors. It can bind to advanced glycation end products (AGEs), generating oxidative stress, activating a variety of cellular signaling channels, causing pro-inflammatory and pro-coagulant responses, and thus causing damage to the vascular endothelium and hematopathological responses [7, 8]. Endogenously secreted RAGE is produced by selective shearing of RAGE pre-RNA, both of which can be hydrolyzed by extracellular matrix metalloproteinases to form cleaved RAGE [9, 10]. Soluble RAGE (sRAGE) includes Endogenously secreted RAGE and cleaved RAGE, which can compete with RAGE for ligands without signaling, inhibit the role of RAGE in disease, and provide protection against CKD [11]. This article aims to study the serum RBP4 and sRAGE levels of CKD patients, observe the correlation between serum RBP4 and sRAGE levels and the condition of CKD, and analyze the diagnostic value of serum RBP4 and sRAGE levels for CKD. The reports are as follows.

## 2. Material and Methods

### 2.1. Normal Information

53 CKD patients diagnosed in our hospital from October 2018 to October 2019 were selected as the observation group, including 32 males and 21 females. The age was 37–81 years, with an average age of (63.28 ± 10.39) years old. The primary diseases included 21 cases of chronic glomerulonephritis, 12 cases of diabetic nephropathy, 8 cases of hypertensive nephropathy, 4 cases of polycystic kidney disease, and 8 cases of other causes. According to GFR, the observation group was divided into 5 subgroups. GFR ≥ 90 (mL/(min·1.73 m^2^)) is the CKD1 group (*n* = 12), 60 ≤ GFR < 90 (mL/(min·1.73 m^2^)) is the CKD2 group (*n* = 10), 30 ≤ GFR < 60 (mL/(min·1.73 m^2^)) is the CKD3 group (*n* = 11), 15 ≤ GFR < 30 (mL/(min·1.73 m^2^)) is the CKD4 group (*n* = 9), and GFR < 15 (mL/(min·1.73 m^2^)) is the CKD5 group (*n* = 11). 53 cases of healthy people who underwent physical examination during the same period were selected as the control group, including 30 males and 23 females. The age was 35–82 years old, with an average age of (62.95 ± 10.27) years old. There was no statistically significant difference between the two groups of general information (*P* > 0.05), and they were comparable. This study was approved by the ethics committee of our hospital, and the patients and family members gave informed consent and signed an informed consent form.

### 2.2. Inclusion Criteria

All comply with the “Guidelines for Screening, Diagnosis, and Prevention of Chronic Kidney Disease”: renal impairment at 3 months and above with/without GFR decline; GFR less than 60 mL/(min·1.73 m^2^) at 3 months and above with/without manifestation of renal impairment; no acute deterioration of renal function; no mental and cognitive impairment; and patients with a higher degree of cooperation.

### 2.3. Exclusion Criteria

Patients with combined renal stone, renal tuberculosis, and renal cystic disease; patients with peritoneal dialysis and surgical trauma; patients with combined serious cardiovascular disease, hematological system disease, immune system disease, and malignant tumor; patients with combined pregnancy and thyroid abnormalities; and patients with drug or toxic poisoning.

### 2.4. Research Method

Five milliliters of venous blood was drawn from the two groups on an empty stomach for future testing. Centrifuge at 3000 r/min for 10 min to take the supernatant and store it in the refrigerator at −80°C for inspection. The enzyme-linked immunosorbent assay was used to detect serum RBP4 and sRAGE. The enzymatic measurement was used to detect serum creatinine (Scr). The kit was purchased from Beijing Biolab Technology Co., Ltd., and the operation was carried out in strict accordance with the kit instructions. The eGFR was estimated using the modification of diet in renal disease (MDRD) formula. The MDRD formula is as follows: eGFR (ml/min·1.73 m^2^) = 186 × (Scr/88.4) − 1.154×(age) − 0.203 × (0.742 female).

### 2.5. Statistical Methods

The results of this experiment were statistically analyzed by SPSS 20.0. Count data were expressed by (rate), and chi-square test was used for their comparison between groups. Measurement data were expressed by (mean ± standard deviation), and *t*-test was used for their comparison between groups; one-way analysis of variance and LSD post hoc test were used for comparisons between multiple groups. Correlation analysis adopts Pearson correlation analysis. The receiver operating characteristic curve (ROC) was drawn, and the area under the ROC curve (AUC) was used to evaluate the diagnostic value. *P* < 0.05 indicates that the difference is statistically significant.

## 3. Results

### 3.1. Comparison of Serum RBP4 and sRAGE Levels between the Two Groups

The serum RBP4 levels of the control group and the observation group were (38.59 ± 16.84) and (173.51 ± 58.67) mg/L, respectively. The serum sRAGE levels of the control group and the observation group were (0.81 ± 0.47) and (0.52 ± 0.23) ng/mL, respectively. The serum RBP4 level of the observation group was higher than that of the control group, and the serum sRAGE level was lower than that of the control group, and the differences were statistically significant (*P* <  0.05), as shown in Figure 1.

### 3.2. Comparison of Serum RBP4 and sRAGE Levels in CKD Patients of Different Stages

The serum RBP4 levels of the CKD1 group, the CKD2 group, the CKD3 group, the CKD4 group, and the CKD5 group were (48.65 ± 17.36), (82.49 ± 22.58), (148.05 ± 40.32), (207.14 ± 32.27), and (334.06 ± 36.31) mg/L, respectively. The serum sRAGE levels of the CKD1 group, the CKD2 group, the CKD3 group, the CKD4 group, and the CKD5 group were (0.95 ± 0.28), (0.71 ± 0.23), (0.54 ± 0.16), (0.41 ± 0.10), and (0.30 ± 0.11) ng/mL, respectively. With the progress of CKD, the serum RBP4 level of patients increased, and the serum sRAGE level decreased; the difference was statistically significant (*P* < 0.05), as shown in Figure 2.

### 3.3. Correlation Analysis of Serum RBP4 and sRAGE Levels in Observation Group and CKD Condition

The results of Pearson correlation analysis showed that the serum RBP4 level in the observation group was negatively correlated with GFR (*r* = −0.661, *P* < 0.001), that is, it was positively correlated with the condition of CKD; serum sRAGE level was positively correlated with GFR (*r* = 0.524, *P* = 0.019), that is, it was negatively correlated with the condition of CKD, as shown in Figure 3.

### 3.4. Diagnostic Value of Serum RBP4 and sRAGE and Combined Diagnosis for the Condition of CKD

The AUC of serum RBP4 diagnosis for the condition of CKD was 0.788 (95% CI 0.675–0.901). When the best cutoff value was 0.509, the sensitivity was 68.8% and the specificity was 82.1%; the AUC of serum sRAGE diagnosis for the condition of CKD was 0.773 (95% CI 0.656–0.890); when the best cutoff value was 0.714, the sensitivity was 28.6% and the specificity was 56.7%; the AUC of the combined diagnosis for the condition of CKD by the two indicators was 0.898 (95% CI 0.821–0.976). When the best cutoff value was 0.761, the sensitivity was 87.5% and the specificity was 88.6%, as shown in Table 1 and Figure 4.

## 4. Discussion

According to incomplete reports, due to factors such as increasing population aging and changes in lifestyles, the prevalence of CKD in China has reached about 10%, which is becoming another important threat to human health after cardiovascular and cerebrovascular diseases, tumors, and diabetes [12]. In addition, according to epidemiological research studies, CKD is an independent risk factor for cardiovascular disease, and the incidence of cardiovascular disease in patients has increased significantly before the progression of CKD to uremia, thus making it a serious public health problem in today's society [13, 14]. Prior to CKD stage III, patients may be asymptomatic or experience only mild discomfort [15–17]. However, when the disease continues to progress until the GFR drops below 15 mL/(min·1.73 m^2^), it suggests that the disease has progressed to the ESRD stage. The renal function of ESRD patients is significantly lower than that of healthy people, which seriously affects the quality of life of patients and even threatens the lives of patients [18]. Therefore, how to detect DN early and give appropriate treatment in time is extremely important. Maintenance hemodialysis (MHD), abdominal dialysis, and kidney transplantation are the main alternative treatments for ESRD patients. Among them, MHD performs substance exchange by draining blood from the body to the dialyzer outside the body to remove metabolic waste from the body, maintain electrolyte balance, maintain acid-base balance, and remove excess water in the body [19, 20]. RBP4 is a small-molecular-weight protein and a transporter of retinol in the blood. It can be used as a marker for many diseases. It is often present in the blood as a complex. The decomposed and free RBP4 is mostly absorbed and decomposed by the renal tubules after being filtered by the glomeruli [21–23]. RAGE is a multi-ligand transmembrane signal transduction receptor circulating in human blood. Due to the diversity of RAGE ligands, RAGE can participate in various pathological processes such as atherosclerosis, tumor formation, and kidney disease by activating different intracellular signaling pathways. sRAGE is a decoy receptor for RAGE ligands, which can compete with RAGE for binding ligands, thereby inhibiting the progression of RAGE-related pathological processes [24–26]. sRAGE is mainly derived from endothelial cells, has no transmembrane and intracellular segments, and contains a ligand-binding region, which can compete with RAGE for ligand binding, thereby inhibiting the progression of RAGE-related pathological processes and protecting CKD patients [27–29].

The results of this study showed that the serum RBP4 level of the observation group was higher than that of the control group, and the serum sRAGE level was lower than that of the control group. With the progress of CKD, the patient's serum RBP4 level increased, and the serum sRAGE level decreased. The reason is that the kidney is the main place where RBP4 is metabolized in the body. RBP4 in the human body is filtered by the glomerulus and then absorbed by the renal tubules. Renal function damage will lead to an increase in the level of RBP4 [30]. In addition, RBP4 can interfere with the insulin receptor signaling pathway, thereby affecting the body's insulin resistance. Elevated levels of RBP4 will lead to increased human insulin resistance, which in turn will increase the incidence of diabetic nephropathy, which is one of the main secondary factors of CKD [31]. RAGE can combine with AGEs to trigger oxidative stress and form a large amount of reactive oxygen species. Active oxygen can activate phosphatidylinositol signaling pathway and mitogen-activated protein kinase signaling pathway, so that nuclear factor-κB and activator protein 1 are phosphorylated and activated, and then regulate the transcription of corresponding genes, resulting in the increase of growth factors and extracellular matrix, and finally the formation of glomerulosclerosis and renal function injury take place. sRAGE is a decoy receptor for AGEs, can compete with RAGE to bind to AGEs, and can inhibit the renal function damage process mediated by AGE-RAGE signaling pathway [32–34]. Therefore, the serum RBP4 level was positively correlated with the condition of CKD, and the serum sRAGE level was negatively correlated with the condition of CKD.

ROC curve results showed that the AUC of serum RBP4 combined with serum sRAGE to diagnose the condition of CKD patients was higher than that of serum RBP4 and serum sRAGE alone to diagnose the condition of CKD patients. It shows that serum RBP4 and sRAGE levels have certain reference significance for the diagnosis of CKD patients, and the diagnostic value of combined diagnosis is significantly higher than that of a single index. The reason is that the ability of the kidneys of CKD patients to filter and remove small molecule proteins is reduced, which leads to a significant increase in the content of RBP4 in the serum [35]. The increase of RBP4 level is a positive feedback signal of the body, which can increase the release of RBP4 complex from the liver. Therefore, when the glomerular filtration function decreases, it further increases the serum RBP4 level [36, 37]. When the proximal tubules of CKD patients are injured, the significant increase in urine RBP4 level is a sensitive indicator reflecting the damage of the proximal tubules. RAGE can be expressed in conjunction with AGEs to trigger oxidative stress response, regulate the transcription of corresponding genes, and cause damage to the vasculature and renal function. sRAGE can inhibit the damage of RAGE to the patient's kidney and the damage to the vasculature by competitively binding AGEs, which is a protective factor for patients. Detection of serum sRAGE levels in patients can effectively diagnose CKD [38, 39]. The production of RBP4 is not constant, and the combination of serum RBP4 and sRAGE can improve the diagnostic value of CKD [40].

## 5. Conclusion

In patients with CKD, serum RBP4 level increased and serum sRAGE level decreased. The results of the study showed that serum RBP4 and serum sRAGE were closely related to the condition of CKD. Serum RBP4 combined with sRAGE has a high diagnostic value for the condition of CKD, which is worthy of clinical application. Nevertheless, there are some defects such as the small sample size, which may affect the results. The specific mechanism of serum RBP4 on renal damage in CKD patients has not been further elucidated, and further research is needed in the future.

## Figures and Tables

**Figure 1:** Serum RBP4 and sRAGE levels in the two groups. (a) The level of serum RBP4 in the 2 groups ($\bar{x}$ ± *s*, mg/L). (b) The level of serum sRAGE in the two groups ($\bar{x}$ ± *s*, ng/mL). Note: ^*∗*^*P* < 0.05, compared with control group.

**Figure 2:** Comparison of serum RBP4 and sRAGE levels in patients with different degrees of CKD. (a) The level of serum RBP4 in the 5 groups ($\bar{x}$ ± *s*, mg/L). (b) The level of serum sRAGE in the 5 groups ($\bar{x}$±*s*, ng/mL). Note: ^*∗*^*P* < 0.05, compared with CKD1 group; ^#^*P* < 0.05, compared with CKD2 group; ^^^*P*<0.05, compared with CKD3 group; ^&^*P* < 0.05, compared with CKD4 group.

**Figure 3:** Correlation between serum RBP4 and sRAGE levels and the condition of CKD. (a) Correlation between serum RBP4 level and the condition of CKD (GFR). (b) Correlation between serum sRAGE level and the condition of CKD (GFR).

**Figure 4:** The diagnostic value of serum RBP4 and sRAGE and combined diagnosis for the condition of CKD. (a) The diagnostic value of serum RBP4 for the condition of CKD. (b) The diagnostic value of serum sRAGE for the condition of CKD. (c) The diagnostic value of serum RBP4 combined with sRAGE for the condition of CKD.

**Table 1:** The diagnostic value of serum RBP4 and sRAGE and combined diagnosis for CKD.

Diagnostic indexes	AUC	95% CI	Cutoff value	Sensitivity (%)	Specificity (%)
RBP4	0.788	0.675–0.901	0.509	68.8	82.1
sRAGE	0.773	0.656–0.890	0.714	28.6	56.7
Combined diagnosis	0.898	0.821–0.976	0.761	87.5	88.6

## Data Availability

The data used and/or analyzed in the current research can be obtained from the corresponding author upon reasonable request.

## References

[1] Mallappallil M. C., Fishbane S., Wanchoo R., Lerma E., Roche-Recinos A., Salifu M. (2018). Practice patterns in transitioning patients from chronic kidney disease to dialysis: a survey of United States nephrologists. *BMC Nephrology*.

[2] Wanner C., Herzog C. A., Turakhia M. P. (2018). Chronic kidney disease and arrhythmias: highlights from a kidney disease: improving global outcomes (KDIGO) controversies conference. *Kidney International*.

[3] Kim S. M., Song I. H. (2018). Hepatitis C virus infection in chronic kidney disease: paradigm shift in management. *The Korean Journal of Internal Medicine*.

[4] Morfin-Otero R., Garza-Gonzalez E., Garcia G. G. (2018). *Clostridium difficile* infection in patients with chronic kidney disease in Mexico. *Clinical Nephrology*.

[5] Aggarwal A., Gupta R., Negi V. S. (2017). Urinary haptoglobin, alpha-1 anti-chymotrypsin and retinol binding protein identified by proteomics as potential biomarkers for lupus nephritis. *Clinical and Experimental Immunology*.

[6] Norden A. G. W., Burling K. A., Zeni L., Unwin R. J. (2019). A new estimate of the glomerular sieving coefficient for retinol-binding protein 4 suggests it is not freely filtered. *Kidney International Reports*.

[7] Belmokhtar K., Ortillon J., Jaisson S. (2019). Receptor for advanced glycation end products: a key molecule in the genesis of chronic kidney disease vascular calcification and a potential modulator of sodium phosphate co-transporter PIT-1 expression. *Nephrology Dialysis Transplantation*.

[8] Rabbani N., Thornalley P. J. (2018). Advanced glycation end products in the pathogenesis of chronic kidney disease. *Kidney International*.

[9] Liu B.-C., Tang T.-T., Lv L.-L., Lan H.-Y. (2018). Renal tubule injury: a driving force toward chronic kidney disease. *Kidney International*.

[10] Vanholder R., Gryp T., Glorieux G. (2018). Urea and chronic kidney disease: the comeback of the century? (in uraemia research). *Nephrology Dialysis Transplantation*.

[11] Rebholz C. M., Astor B. C., Grams M. E. (2015). Association of plasma levels of soluble receptor for advanced glycation end products and risk of kidney disease: the Atherosclerosis Risk in Communities study. *Nephrology Dialysis Transplantation*.

[12] Bundy J. D., Chen J., Yang W. (2018). Risk factors for progression of coronary artery calcification in patients with chronic kidney disease: the CRIC study. *Atherosclerosis*.

[13] Mafham M. M., Staplin N., Emberson J. (2018). Prognostic utility of estimated albumin excretion rate in chronic kidney disease: results from the Study of Heart and Renal Protection. *Nephrology Dialysis Transplantation: Official Publication of the European Dialysis and Transplant Association-European Renal Association*.

[14] Zhang L., Wang Z., Chen Y. (2018). Prevalence and risk factors associated with chronic kidney disease in adults living in 3 different altitude regions in the Tibetan Plateau. *Clinica Chimica Acta*.

[15] Liu X., Zhai T., Ma R., Luo C., Wang H., Liu L. (2018). Effects of uric acid-lowering therapy on the progression of chronic kidney disease: a systematic review and meta-analysis. *Renal Failure*.

[16] Di Iorio B. R., Bellasi A., Raphael A. (2020). Correction to: treatment of metabolic acidosis with sodium bicarbonate delays progression of chronic kidney disease: the UBI Study. *Journal of Nephrology*.

[17] Clark W. F., Sontrop J. M., Huang S.-H. (2018). Effect of coaching to increase water intake on kidney function decline in adults with chronic kidney disease. *Journal of the American Medical Association*.

[18] Sowtali S., Harith S., Mohd Shah A. (2020). Educational needs of chronic kidney disease patients who presented to tengku ampuan afzan hospital: preliminary findings. *Saudi Journal of Kidney Diseases and Transplantation*.

[19] Schiff R., Freill H. (2020). Improving access to phosphorus- and sodium-restricted foods for people living with chronic kidney disease in remote First Nations. *Rural and Remote Health*.

[20] Kalaitzidis R. G., Elisaf M. S. (2018). Treatment of hypertension in chronic kidney disease. *Current Hypertension Reports*.

[21] Amiri M., Ramezani Tehrani F., Amanollahi Soudmand S., Behboudi‐Gandevani S., Sabet Z., Azizi F. (2020). Low serum testosterone levels and the incidence of chronic kidney disease among male adults: a prospective population‐based study. *Andrology*.

[22] Wang X., Huang Y., Gao J., Sun H., Jayachandran M., Qu S. (2020). Changes of serum retinol-binding protein 4 associated with improved insulin resistance after laparoscopic sleeve gastrectomy in Chinese obese patients. *Diabetology & Metabolic Syndrome*.

[23] Wang X., Chen X., Zhang H. (2020). Circulating retinol-binding protein 4 is associated with the development and regression of non-alcoholic fatty liver disease. *Diabetes and Metabolism*.

[24] Fukami K., Taguchi K., Yamagishi S.-i., Okuda S. (2015). Receptor for advanced glycation endproducts and progressive kidney disease. *Current Opinion in Nephrology and Hypertension*.

[25] Elmhiri G., Mahmood D. F. D., Niquet-Leridon C. (2015). Formula-derived advanced glycation end products are involved in the development of long-term inflammation and oxidative stress in kidney of IUGR piglets. *Molecular Nutrition & Food Research*.

[26] Lee E. J., Park E. Y., Mun H. (2015). Soluble receptor for advanced glycation end products inhibits disease progression in autosomal dominant polycystic kidney disease by down-regulating cell proliferation. *The FASEB Journal*.

[27] Sun H., Yuan Y., Sun Z. (2016). Update on mechanisms of renal tubule injury caused by advanced glycation end products. *BioMed Research International*.

[28] Yuan Y., Sun H., Sun Z. (2017). Advanced glycation end products (AGEs) increase renal lipid accumulation: a pathogenic factor of diabetic nephropathy (DN). *Lipids in Health and Disease*.

[29] Chang J.-T., Liang Y.-J., Hsu C.-Y. (2017). Glucagon-like peptide receptor agonists attenuate advanced glycation end products-induced inflammation in rat mesangial cells. *BMC Pharmacology and Toxicology*.

[30] Li G., Esangbedo I. C., Xu L. (2018). Childhood retinol-binding protein 4 (RBP4) levels predicting the 10-year risk of insulin resistance and metabolic syndrome: the BCAMS study. *Cardiovascular Diabetology*.

[31] Wang F., Cao G., Liu Q., Li X, Song M, Zhang Z (2018). Retinol-binding protein 4 regulates the biological functions and molecular mechanisms of JEG-3 cells. *International Journal of Clinical and Experimental Pathology*.

[32] Al-Qattan K. K., Mansour M. H., Thomson M., Ali M. (2016). Garlic decreases liver and kidney receptor for advanced glycation end products expression in experimental diabetes. *Pathophysiology*.

[33] Brinkley T. E., Leng X., Nicklas B. J. (2017). Racial differences in circulating levels of the soluble receptor for advanced glycation endproducts in middle-aged and older adults. *Metabolism*.

[34] Thomas M. C., Woodward M., Neal B. (2015). Relationship between levels of advanced glycation end products and their soluble receptor and adverse outcomes in adults with type 2 diabetes. *Diabetes Care*.

[35] Fan J., Yin S., Lin D. (2019). Association of serum retinol-binding protein 4 levels and the risk of incident type 2 diabetes in subjects with prediabetes. *Diabetes Care*.

[36] Du C., Kong F. (2019). A prospective study of maternal plasma concentrations of retinol-binding protein 4 and risk of gestational diabetes mellitus. *Annals of Nutrition and Metabolism*.

[37] Kieneker L. M., Hartmann O., Bergmann A. (2018). Proenkephalin and risk of developing chronic kidney disease: the Prevention of Renal and Vascular End-stage Disease study. *Biomarkers*.

[38] Ruelas Cinco E. D. C., Ruíz Madrigal B., Domínguez Rosales J. A. (2019). Expression of the receptor of advanced glycation end-products (RAGE) and membranal location in peripheral blood mononuclear cells (PBMC) in obesity and insulin resistance. *Iranian Journal of Basic Medical Sciences*.

[39] Cheng Y.-Z., Yang S.-L., Wang J.-Y. (2018). Irbesartan attenuates advanced glycation end products-mediated damage in diabetes-associated osteoporosis through the AGEs/RAGE pathway. *Life Sciences*.

[40] Stenvinkel P., Painer J., Kuro-O M. (2018). Novel treatment strategies for chronic kidney disease: insights from the animal kingdom. *Nature Reviews Nephrology*.

